# A Mobile Application Penyikang Applied in Postpartum Pelvic Floor Dysfunction: A Cross-Sectional Study to Analyze the Factors Influencing Postpartum Pelvic Floor Muscle Strength and Women's Participation in Treatment

**DOI:** 10.1155/2020/4218371

**Published:** 2020-07-28

**Authors:** Juan Li, Xiaoyan Sun, Congyu Wang, Zujuan Zhang, Zhenwei Xie

**Affiliations:** ^1^Women's Hospital, Zhejiang University School of Medicine, Hangzhou, Zhejiang, China; ^2^Department of Psychology, Tsinghua University, Beijing, China

## Abstract

**Objectives:**

Postpartum pelvic floor muscle (PFM) injuries are the result of pregnancy and delivery, which lead to a series of symptoms requiring long-term follow-up. Mobile health platforms are progressively used for monitoring clinical conditions in medical subjects. This survey was a cross-sectional design based on collecting data from an application (Penyikang). We retrospectively analyzed the risk factors for weak postpartum PFM and further analyzed the factors influencing women's participation in the treatment which may help to improve the app's application in the future.

**Methods:**

We enrolled postpartum women who gave birth at the Women's Hospital, Zhejiang University School of Medicine from August to November 2017; trained them to use the app; and collected the demographic and clinical information. This app requires users to fill questionnaires to assess their knowledge of pelvic floor dysfunction (PFD) and pelvic floor muscle training (PFMT) and experience with PFMT, and each therapy evaluation was restored. The relationship between the knowledge of PFMT/PFD, UI symptoms, and PFM strength was analyzed. Cluster analysis was used to define the degree of participation and identify the factors influencing the patients' participation in intensive therapy and evaluation.

**Results:**

1982 postpartum women who enrolled in the app program were defined as weak PFM. Younger maternal age, cesarean section, and without delivery injury were found as the prognostic factors to PFM strength (both type I and type II muscle fibers) (*P* < 0.05), and higher educational level was also in favor of type II muscle fibers (*P* < 0.05). Patient-reported UI symptoms were associated with weak PFM strength (*P* < 0.05); there were no significant differences between knowledge of PFMT or PDF and PFM strength. Finally, patients with a higher degree of participation were more likely to accept the treatment (*P* < 0.05).

**Conclusions:**

The mobile app provides a new applicative way to investigate postpartum PFD. The factors influencing women's participation can help us focus on strategies to increase the patients' compliance, and then we will apply the app into more areas to improve the prevention and treatment of postpartum PFD.

## 1. Introduction

Urinary incontinence (UI), which is regarded as one type of pelvic floor dysfunction (PFD), often is complicated by pelvic organ prolapse (POP). UI has a high incidence rate with one in three women, and the quality of life of the patients may be affected during their lifetime [1–3]. Vaginal delivery is regarded as a predominant and independent risk factor for PFD [2, 3]. Furthermore, the prevalence of UI is increasing over time [4]; therefore, we have to admit that the prevention of postpartum UI is becoming a challenging and long-term task in the field of gynaecology and obstetrics.

Pelvic floor muscle (PFM) strength was impaired in women who suffered from PFD [5], and it may subsequently lead to UI, POP, and fecal incontinence [6]. The scale of PFM strength has been reported to be correlated with PFDs of women at postpartum 6 to 8 weeks [7]. Pelvic floor muscle training (PFMT) is recommended as one of the first-line methods for the treatment of PFD [8, 9], and it can improve the condition of PFD in about two-thirds of patients [10]. Recent Cochrane reviews support the recommendation of PFMT to women with UI [8], but these benefits are not yet firmly confirmed for POP [9]. Despite the benefits, women suffering from UI rarely seek treatment because of privacy issue or lack of knowledge of the disease severity. Since PFD has become a global health issue, we need to find an effective and easily accessible method to motivate people to strengthen their cognition of disease and participate in the treatment of the disease.

Nowadays, internet and phone apps bring benefits and information to patients especially those suffering from chronic diseases [11]. The Web easily broadcasts the information to the public timely and effectively [12]. Several studies have demonstrated that mobile health technology can improve clinical outcomes [13–15], even better than traditional nursing intervention [16]. The application of apps also significantly improved the therapy-adherence rates [17]. UI is a chronic disease but lacks management, and apps may help the patients get access to more information on PFD, acquire their personal evaluation results, and contact doctors anytime and anywhere instead of the traditional out-patient follow-up. Therefore, we designed a mobile app named Penyikang aimed at inviting postpartum women to participate in the follow-up program, helping them to get a better understanding of PFD, and improving their willingness to participate in and adhere to PFMT. This survey was a cross-sectional design wherein we first identified the risk factors for weak postpartum PFM strength and the association between weak PFM strength and UI symptoms. Moreover, we believe women's knowledge of PFD and symptoms may play crucial roles in women's willingness to receive the instructions on disease prevention and therapy.

## 2. Materials and Method

### 2.1. App Program

Penyikang is an iOS/Android app developed by designers and engineers on the basis of theories and evidence, as well as the needs of users. It facilitates postpartum women to get access to PFD information, their evaluation, and the clinical outcomes and allows them to consult with the doctors if they have problems anytime. At the time of development, the company tested the prototype of Penyikang with experts with different backgrounds and revised iteratively to improve its usability and utility. The assistants introduced Penyikang to postpartum women who then voluntarily installed the app and filled up the demography form with informed consent. The related delivery and evaluation synchronous data will be transmitted to the app when they come to the hospital for routine six-week postpartum out-patient follow-up.

The assistants helped the enrolled patients install the app on their smartphones and instructed them on how to use the app. The doctors can capture, review, and analyze the data and analyze the factors influencing postpartum PFD or other information. The app collected and stored personal data much easier and could motivate patients to participate in the program, so that it makes the whole follow-up process more convenient and retrospective.

### 2.2. Clinical Information of the Patients

The study protocol was approved by the institutional review board of Women's Hospital, Zhejiang University School of Medicine. Due to time and budget restrictions, we retrospectively identified postpartum women over a 4-month recruitment period (August to November 2017). Women 18 years and older who gave birth after 37 weeks gestation were eligible. Based on the preliminary findings, we estimated that 650-700 women would be enough to determine the risk factors. Since a response rate of 35% of women was considered possible and reasonable, approximately 1700-2000 women should be recruited.

At routine six weeks of postpartum control, postpartum women were recruited to fill the basic individual information and complete questionnaires on the app. Meanwhile, they were evaluated for PFM strength.

The International Consultation on Incontinence Questionnaire-Urinary Incontinence Short Form (ICIQ-UI SF) was used to evaluate UI severity. The questionnaire regarding knowledge of PFD was designed with several questions to assess their knowledge, awareness of the symptoms, and its influence on their lives. The questionnaire about knowledge of PFMT reflected their desire to seek methods to solve the problem and the awareness that PFMT is an effective way.

Women's PFM strength was evaluated by a validated method and classified by the Oxford scale [18]. The details were shown in Table 1. Pelvic floor muscle strength was considered abnormal if both type I (the fibers that produce low-intensity as well as long-duration movements of the muscle) and II muscle fibers (the fibers that produce high-intensity as well as short-duration movements of the muscle) received a score [5] less than grade 3; it was measured in the participating postpartum women on 6–8 weeks after delivery by two experienced physiotherapists following the protocol [19] to reduce detection bias.

Of the total 2109 postpartum women attending the app program, 739 completed the questionnaire covering UI symptoms, 778 responded to the questionnaire of knowledge of PFD, and 739 responded to the questionnaire of knowledge of PFMT. The response rate was 35.04%, 36.89%, and 35.04%, respectively. The nonresponse rates of the study were higher than we expected; thus, we performed a comparative analysis between women included in the final sample and those who quit the study. We found that the homogeneity of both groups suggested that the effect of the loss did not greatly influence the results of the final response samples. In this survey, all the respondents were not promised any benefits or feedback, and no incentives were offered, either.

### 2.3. Data Analysis

The outcome results are frequencies and percentages which are reported for categorical data. Forward selection and backward elimination techniques were used to find the final regression model. Shapiro–Wilk tests were used to measure the normality of distributions in variables.

Linear discriminant analysis was performed to introduce multiple logistic regression analysis to define risk factors for the weak PFM strength using list-wise deletion of cases with missing data, and adjusted odds ratios (ORs) and their 95% confidence intervals (CIs) were calculated. The x^2^ test was used for evaluating nominal variables, and differences among groups for ordinal variables were evaluated by Kruskal-Wallis variance analysis. When the *P* value from the Kruskal-Wallis test statistic was statistically significant, then a multiple comparison test was performed to determine which groups differed from which other groups. In our study, the above-mentioned calculations were used to investigate the association between knowledge of PFD/PFMT and PFM strength. We used cluster analysis to classify the degree of participation, and the x^2^ test and Kruskal-Wallis test were also performed to analyze the characteristic difference from high or low degree of participation. *P* values less than 0.05 were considered significant. SPSS 21 (Armonk, NY: IBM Corp.) was used for analysis.

## 3. Results

### 3.1. Construction and Validation of the App

Penyikang was developed by a professional obstetrician, gynaecologists, and engineers on the basis of theories and evidence, as well as the needs of users. Before developing the app, the obstetrician and gynaecologists performed literature research and found that PFM strength is strongly associated with the development of PFD, and PFMT is recommended as the first-line treatment of PFD in the postpartum period. Moreover, other components, for example, knowledge of PFD, knowledge of PFMT, and the concept of UI, were also decided as part of the content to be included in the app. At the time of development, the company tested a prototype of Penyikang with experts with different backgrounds and revised iteratively to improve its usability and utility.  Figure 1 shows the system architecture.

When app was developed, the assistants introduced Penyikang to postpartum women who then voluntarily installed the app and filled up the demography form with informed consent.  Figure 2 presents the major working interface of Penyikang:

- When postpartum women first use Penyikang, they will receive an alert message that they should come to the hospital for routine postpartum follow-up
- Main interface of Penyikang
- Postpartum women are required to fill their basic individual information and complete questionnaires on the app; the synchronous delivery data will be transmitted to the app
- List of experts from which patients can consult a doctor online when they have problems

Next, the related delivery and evaluation synchronous data will be transmitted to the app when they come to the hospital for routine six-week postpartum out-patient follow-up (Figure 3).

### 3.2. Association between Characteristics of Participants and Weak Pelvic Floor Muscle Strength

Table 2 shows an overview of relevant demographic and clinical characteristics, and 1982 postpartum women were with weak PFM strength. The preliminary finding was the identification of risk factors for weak PFM strength in postpartum women. The final regression model includes three statistically significant predictors for the risk factors for the strength of type I pelvic floor muscle fibers: maternal age, pelvic floor injuries, and modes of delivery (Table 3). Maternal age less than 35 years old had better type I PFM strength than the elder group, OR = 3.074 (x^2^ = 4.638, *P* < 0.05). Cesarean section seems to be a better protective delivery type for type I PFM strength, OR = 2.581 (x^2^ = 9.683, *P* < 0.05), while we found no delivery injury could better protect the strength of type I muscle fibers, OR = 2.702 (*χ*^2^ = 8.227, *P* < 0.05).

There were strong correlations between the strength of type II pelvic floor muscle fibers and the prognostic factors for PFM strength (*P* < 0.05: educational level, maternal age, pelvic floor injuries, and modes of delivery (Table 4)). Maternal age less than 35 years old, cesarean section, and no delivery injury had better type II pelvic floor muscle strength [OR = 2.956 (x^2^ = 4.537, *P* < 0.05), OR = 2.591 (*χ*^2^ = 9.669, *P* < 0.05), and OR = 2.223 (*χ*^2^ = 5.286, *P* < 0.05), respectively]. Patients who have bachelor degrees had better strength of type II muscle fibers than those who only have high school degrees, OR = 1.795 (*P* < 0.05).

### 3.3. Association of Awareness of UI Symptoms, Knowledge of PFD/PFMT, and Weak Pelvic Floor Muscle Strength

We found that awareness of the UI symptom during pregnancy had a negative correlation with the weak PFM strength (rs (type I muscle fibers) = −0.105, *P* < 0.05; rs (type II muscle fibers) = −0.079, *P* < 0.05). Meanwhile, postpartum UI symptoms, UI severity, UI type or the patients' UI diagnosis by a physician, anal incontinence (AI), and POP were barely associated with weak PFM strength (Table 5).

The questionnaires regarding the patients' knowledge of PFD and PFMT were used, and patients who got the higher scores meant they had a better understanding of PFD or PFMT and their impacts on quality of life. We found that there was no association between knowledge of pelvic floor dysfunction/pelvic floor muscle training and pelvic floor strength (Table 5).

### 3.4. Degree of Participation

A total of 745 postpartum women who used the app came to our hospital for the assessment and therapy. We retrieved and calculated the data by cluster analysis and we defined the high degree of participation as patients followed the pattern of evaluation and PFMT exercise at least 15 times, while the low degree of participation group finished less than 6 times (Table 6). 483 women had a relatively high degree of participation, while 262 women were identified as low-degree participators. We found that patients who were more likely to participate in the app program were often older than the group with low degree of participation (*P* = 0.012), and they were also more aware of the PFD condition (*P* = 0.000) (Table 7).

Results of Table 8 demonstrated that when the patients complain of urine leakage symptoms, during pregnancy or after delivery, they were also more likely to follow this program (*P* = 0.007). On the other hand, the complaints on POP symptoms or sexual dysfunction did not affect their willingness to participate in the program.

## 4. Discussion

In recent years, with growing requirements for a high-quality life, people are more likely to seek help and acknowledge that they should be more concerned over PFD due to its harm and embarrassment. As we know, PFD is preventative and women have a great risk to suffer from postpartum PFD; our goal is to establish good management and a follow-up system. Therefore, we designed the mobile app follow-up system not just to focus on finding the risk factors and/or prognostic factors for PFD but also to inform on the benefits of awareness of PFD and to find strategies to motivate patients to participate in and adhere to evaluation and therapy.

The app Penyikang collected the data about the patients' complaints of PFD, symptoms and delivery information, therapy, and participation evaluation. The results demonstrated that with the app to build up the beneficial follow-up pattern, we have a considerable amount of data about postpartum women attending to find out the risk factors for weak PFM strength. As maternal age over 35 years old led to weaker PFM strength (both type I and II pelvic muscle fibers), younger age could be a protective factor. Women who did not get pelvic floor injuries or experienced cesarean section could get better PFM strength than women who got other types of pelvic floor injuries or modes of delivery. For type II pelvic muscle fibers, the higher education level also seems to be a protective factor. It is easy to understand why patients who are more educated can be more aware of their symptoms and disease prevention. But the results hardly explain why it cannot apply in type I pelvic muscle fibers. The results of impairing PFM strength are similar to other papers' conclusions [18, 20–22]. Nevertheless, some researchers reported PFM strength did not change significantly during pregnancy or after delivery [23].

To our knowledge, the app Penyikang is the first mobile phone-based program conducting the follow-up of postpartum PFD patients and helping them participate in the evaluation and treatment of the disease in China. Since PFD has become a highly prevalent health issue, we are eager to find a way by which patients are willing to follow the pattern and give feedback. It is important to explore the characteristics of active postnatal participants. We analyzed the degree of participation and its correlation with age, educational level, knowledge of PFD, UI symptoms, sexual dysfunction, and prolapse symptoms of the patients. The finding outlined that patients with older age would participate in PFMT and follow-up more actively; meanwhile, they maybe more capable of realizing their suffering from the UI symptoms. When patients had obvious UI symptoms, they were more willing to participate, which was consistent with the results from a survey conducted before [24]. We hope that our work can be dedicated to finding the potential participants, decreasing the morbidity of postpartum PFD, and helping the patients find more appropriate treatments in case they think it is not regarded as an ailment or disease or are uncomfortable to see a doctor. The study allowed further refinement of Penyikang which should be conducted, and it will be useful for public health experts and researchers to improve user-centered mobile Web apps. The mobile app follow-up management program will be prospective as we will introduce it to more areas to prevent the postpartum PFD.

The present work has limitations. First, the app just started working and came into service for a short time and is limited to our hospital, and the average age, educational levels, and others represented were limited to Zhejiang province, China. Differences in the education system and peripartum care between different provinces and cities may reduce generalizability, so we need to introduce the app into more areas to illustrate acute outcomes, and it is still a long-term work. However, a potential limitation is that questions about past behavior and experiences might be subject to recall bias [25], and data might be biased by missing respondents during the survey. Because of the cross-sectional study, we cannot test for causal relationships but can only examine the statistical associations of the outcomes. In a future study, we will capture more user feedback and the degree of participation to improve our app. In addition, a cohort study comparing the influence on patients' follow-up based on the app and the traditional out-patient follow-up mode needs to be conducted in the future to support our view that the app will bring more convenience. In the following studies, the researchers should investigate the risk factors, and a randomized controlled trial should be designed to confirm the conclusions as well.

## Figures and Tables

**Figure 1:** Penyikang recorded and sent data to the terminal computer, which further connected and restored data in the SQL database; researchers can access the SQL database with specific application requirements and analyze the output data. SQL: standard database language.

**Figure 2:** Major working interface of Penyikang: (a) alert message; (b) main interface of Penyikang; (c) individual information and questionnaires; (d) list of experts.

**Figure 3:** All recruited postpartum women will be introduced to download the mobile app, then they will be asked to fill in their related personal information and a series of questionnaires. The clinical evaluation will be administrated to give the results on whether the patient will be followed up at home or continue to do more therapy and improvement.

**Table 1:** The Oxford classification scale.

Grade 0	No contractions
Grade 1	Flicker of muscular contraction
Grade 2	Low intensity but sustained contraction
Grade 3	Moderate contraction, with an increase in intravaginal pressure, squeezing of fingers, and slight elevation of the vaginal wall
Grade 4	Satisfactory contraction, which pushes against the examiner's fingers, with elevation of the vaginal wall in the direction of the pubic symphysis
Grade 5	Strong contraction, firm compression of the examiner's fingers with positive movement in the direction of the pubic symphysis

**Table 2:** Demographic and clinical characteristics, urogynaecological symptoms, pelvic floor-related complaints, and knowledge of pelvic floor dysfunction/pelvic floor muscle training.

		*N* (%)
*Weak PFM*		*N* = 1982
Age when app first used (yrs)	<25	127 (6.41)
	25-34	1354 (68.31)
	35-44	420 (21.19)
	>45	39 (1.97)
	Missing	42 (2.12)
Educational level	Low	82 (4.14)
	Middle	180 (9.08)
	High	1685 (85.02)
	Missing	35 (1.76)
BMI	<25 normal	1425 (71.90)
	25–30 overweight	313 (15.79)
	≥30 obese	209 (10.55)
	Missing	35 (1.76)
Parity	≤2	1872 (94.45)
	>2	58 (2.93)
	Missing	52 (2.62)
Maternal age	<35	1617 (81.58)
	≥35	348 (17.56)
	Missing	17 (0.86)
Heaviest birth weight (g)	<4000	1685 (85.02)
	≥4000	265 (13.37)
	Missing	32 (1.61)
Modes of delivery	Cesarean section	786 (39.66)
	Vaginal delivery	1078 (54.39)
	Forceps	89 (4.49)
	Missing	29 (1.46)
Number of fetuses delivered	Singleton	1798 (90.72)
	Others	148 (7.47)
	Missing	36 (1.81)
Perineum injury type	None	696 (35.12)
	Rupture	462 (23.31)
	Median episiotomy	98 (4.94)
	Lateral episiotomy	541 (27.3)
	Missing	185 (9.33)
*UI complaints and symptoms*		*N* = 739
UI complaints	Yes	228 (30.85)
	No	511 (69.15)
UI prevalence	Before pregnancy	0 (0)
	During delivery	210 (92.1)
	Postpartum	165 (72.4)
UI severity (ICIQ UI-SF sum score)	1-5 slight	28 (12.28)
	6-12 moderate	37 (16.23)
	13-18 severe	163 (71.49)
	19-21 very severe	0 (0)
UI type	Stress	143 (62.72)
	Urgency	9 (3.95)
	Mixed	3 (1.31)
	Others	73 (32.02)
POP complaints	Yes	94 (12.72)
	No	596 (80.65)
	Missing	49 (6.63)
AI	Yes	35 (4.74)
	No	655 (88.63)
	Missing	49 (6.63)
*Knowledge of PFD*		*N* = 778
	0-2 little	86 (11.05)
	3-6 general	362 (46.53)
	7-9 well	330 (42.42)
*Knowledge of PFMT*		*N* = 739
	0-2 little	224 (30.31)
	3-6 general	374 (50.61)
	7-9 well	141 (19.08)

*N*: number; %: percentage; PFM: pelvic floor muscle; educational level—low: lower than or equal to middle school degree, middle: high school degree, and high: higher than or equal to bachelor degree; BMI: body mass index; UI: urinary incontinence, complaint of involuntary loss of urine; ICIQ-UI SF: International Consultation on Incontinence Questionnaire-Urinary Incontinence Short Form; POP: pelvic organ prolapse; AI: anal incontinence, complaint of involuntary loss of feces or flatus; PFD: pelvic floor dysfunction; PFMT: pelvic floor muscle training.

**Table 3:** Prognostic factors for pelvic floor strength: association between strength of type I muscle fibers and demographic information of participants.

		*β*	SE	Wald x^2^	*P*	OR (95% CI)
Age when app first used (yrs)	<25	-0.304	1.215	0.062	0.803	0.738 (0.068~7.996)
	25-34	-0.301	1.138	0.070	0.792	0.740 (0.079~6.890)
	35-44	0.934	1.242	0.566	0.452	2.545 (0.233~29.020)
	>45	0a				
Educational level	Low	-0.667	0.510	1.711	0.191	0.513 (0.189~1.394)
	Middle	-0.262	0.302	0.754	0.385	0.770 (0.425~1.391)
	High	0a				
BMI	<25 normal	0.117	0.290	0.164	0.686	1.124 (0.637~1.986)
	25–30 overweight	0.357	0.337	1.123	0.289	1.429 (0.738~2.768)
	≥30 obese	0a				
Parity	≤2	0.723	0.680	1.132	0.287	2.061 (0.544~7.807)
	>2	0a				
Maternal age	<35	1.123	0.519	4.683	0.030^∗^	3.074 (1.112~3.452)
	≥35	0a				
Heaviest birth weight (g)	<4000	0.554	0.350	2.506	0.113	1.740 (0.876~3.452)
	≥4000	0a				
Modes of delivery	Cesarean section	0.948	0.305	9.683	0.002^∗^	2.581 (1.420~4.693)
	Vaginal delivery	0.070	0.318	0.048	0.826	1.07 (0.575~2.002)
	Forceps	0a				
Number of fetuses delivered	Singleton	0.022	0.506	0.002	0.970	1.022 (0.379~2.769)
	Others	0a				
Perineum injury type	None	0.994	0.347	8.227	0.004^∗^	2.702 (1.370~5.328)
	Rupture	-0.039	0.232	0.028	0.866	0.962 (0.611~1.514)
	Median episiotomy	0.235	0.333	0.500	0.479	1.265 (0.660~2.428)
	Lateral episiotomy	0a				

OR: odds ratios; CI: confidence interval; educational level—low: lower than or equal to middle school degree, middle: high school degree, and high: higher than or equal to bachelor degree; BMI: body mass index; every 0a is defined as the calibration standard; ^∗^*P* < 0.05.

**Table 4:** Prognostic factors for pelvic floor strength: association between strength of type II muscle fibers and demographic information of participants.

		*β*	SE	Wald *χ*^2^	*P*	OR (95% CI)
Age when app first used (yrs)	<25	-1.457	1.212	1.444	0.229	0.233 (0.022~2.507)
	25-34	-1.370	1.135	1.459	0.227	0.254 (0.027~2.347)
	35-44	0.036	1.232	0.001	0.977	1.037 (0.093~11.588)
	>45	0a				
Educational level	Low	-0.454	0.508	0.798	0.372	0.635 (0.235~1.719)
	Middle	-0.585	0.302	3.765	0.052^∗^	0.557 (0.309~1.006)
	High	0a				
BMI	<25 normal	0.041	0.291	0.020	0.889	1.042 (0.589~1.844)
	25–30 overweight	0.347	0.339	1.045	0.307	1.415 (0.728~2.751)
	≥30 obese	0a				
Parity	≤2	0.153	0.674	0.051	0.821	1.165 (0.311~4.371)
	>2	0a				
Maternal age	<35	1.084	0.509	4.537	0.033^∗^	2.956 (1.091~8.020)
	≥35	0a				
Heaviest birth weight (g)	<4000	0.304	0.347	0.767	0.381	1.355 (0.687~2.678)
	≥4000	0a				
Modes of delivery	Cesarean section	0.952	0.306	9.669	0.002^∗^	2.591 (1.422~4.716)
	Vaginal delivery	0.083	0.318	0.068	0.794	1.087 (0.583~2.028)
	Forceps	0a				
Number of fetuses delivered	Singleton	0.504	0.507	0.985	0.321	1.655 (0.612~4.473)
	Others	0a				
Perineum injury type	None	0.799	0.347	5.286	0.022^∗^	2.223 (1.125~4.393)
	Rupture	0.062	0.232	0.072	0.788	1.064 (0.675~1.679)
	Median episiotomy	0.764	0.339	5.089	0.024	2.147 (1.105~4.170)
	Lateral episiotomy	0a				

OR: odds ratios; CI: confidence interval; educational level—low: lower than or equal to middle school degree, middle: high school degree, and high: higher than or equal to bachelor degree; BMI: body mass index; every 0a is defined as the calibration standard; ^∗^*P* < 0.05.

**Table 5:** Results of correlation analysis.

	Type I muscle fibers		Type II muscle fibers	
	Spearman correlation coefficient	*P*	Spearman correlation coefficient	*P*
UI self-reported during pregnancy	-0.105	0.005^∗^	-0.079	0.036^∗^
UI self-reported postpartum	-0.032	0.391	-0.026	0.487
UI severity	-0.032	0.722	-0.018	0.778
UI diagnosis	-0.038	0.294	-0.003	0.937
UI type	-0.047	0.202	-0.011	0.776
AI	-0.036	0.340	-0.035	0.342
POP	-0.011	0.764	0.007	0.852
Knowledge of PFD	0.026	0.468	0.047	0.187
Knowledge of PFMT	0.070	0.055	0.063	0.089

UI: urinary incontinence, complaint of involuntary loss of urine; AI: anal incontinence, complaint of involuntary loss of feces or flatus; POP: pelvic organ prolapse; ^∗^*P* < 0.05.

**Table 6:** Cluster analysis to define the degree of participation of treatment (*N* = 745).

	Low degree participation group	High degree participation group
Times of treatments	6	15
*N*	483	262

*N*: number.

**Table 7:** Association between characteristics of participants and the degree of participation.

	*W*		7	*P*
	Low (*n* = 483)	High (*n* = 262)		
Age when app first used	231828.00	275700.00	-2.522	0.012^∗^
Educational level	236986.00	268529.00	-1.757	0.079
Knowledge of PFD	209576.00	274060.00	-3.932	0.000^∗^

*n*: number; low: low degree participation group; high: high degree participation group; PFD: pelvic floor dysfunction. ^∗^*P* < 0.05.

**Table 8:** Association between symptoms of participants and the degree of participation.

*χ* ^2^		*N* (%)			*P*
		Low	High		
Leakage urine	No	297 (51.7)	278 (48.3)	7.304	0.007^∗^
	Yes	186 (43.1)	246 (56.9)		
Sexual dysfunction	No	405 (48.7)	426 (51.3)	1.136	0.287
	Yes	78 (44.3)	98 (55.7)		
POP	No	746 (89.8)	85 (10.2)	1.223	0.269
	Yes	153 (86.9)	23 (13.1)		

*N*: number; %: percentage; low: low degree participation group; high: high degree participation group; POP: pelvic organ prolapse. ^∗^*P* < 0.05.

## Data Availability

Data is available upon request from the corresponding author.
